The article "Renal Doppler Ultrasound in the Evaluation of Renal Function in Patients with Sepsis" was retracted in 2023. Reasons: signs of a paper mill; compromised peer review; unreliable results or conclusions.

# Renal Doppler Ultrasound in the Evaluation of Renal Function in Patients with Sepsis

**DOI:** 10.1155/2022/3472405

**Published:** 2022-04-26

**Authors:** Aili Yu, Qiuhong Zhao, Yimeng Qu, Guohua Liu

**Affiliations:** Department of ICU, Inner Mongolia Xing'anmeng People's Hospital, Ulanhot, 137400 Inner Mongolia, China

## Abstract

This study was aimed to explore the renal Doppler ultrasound in the evaluation of renal function in patients with sepsis. Fifty patients with sepsis or septic shock were classified into the acute kidney injury (AKI) group (n =25) and the non-AKI group (n =25) according to whether they had AKI. The measurements of renal resistance index (RRI) and power Doppler ultrasound (PDU) were performed on all patients within 7 days of admission to the intensive care unit (ICU). The patient's renal function was assessed. The results showed that the RRI of the two groups showed a slight upward trend over time, and the RRI of the AKI group was higher than that of the non-AKI group. After 7 days in AKI group, the areas under the receiver operating characteristic (ROC) curves of RRI were 0.745, 0.683, 0.729, 0.856, 0.793, 0.819, and 0.836 (P <0.05). There were no statistically considerable differences in areas under ROC curves between the two groups (P >0.05). The grouping of AKI and the time were both fixed effects, and the individual patients were randomized effects. Besides, the linear models were statistically analyzed. The results showed that the differences between the two groups were statistically insignificant (P >0.05). There was no significant difference in the PDU scores measured at different times within 7 days after ICU admission between the two groups (P >0.05). In conclusion, renal Doppler ultrasound had a good adoption effect in the evaluation of the renal function of patients with severe sepsis, which is worth promoting in clinical practice.

## 1. Introduction

Acute kidney injury (AKI) is one of the most common problems in critically ill patients in the clinic as well as one of the adverse prognostic factors [1]. AKI can be caused by various factors, such as hypovolemia, shock, major surgery, trauma, and heart failure, of which sepsis is the most common [2]. AKI patients generally need to be admitted to the intensive care unit (ICU). The proportion of renal replacement therapy (RRT) will increase, and the short-term and long-term mortality will increase. It can develop into chronic kidney disease in some patients [3, 4]. In recent years, despite advances in important support and resuscitation techniques, the incidence and mortality of sepsis-associated AKI remain high [5]. When sepsis occurs, pathogens and activated immune cells produce many inflammatory mediators and release them into the blood [6]. The kidney needs to filter out 120-150 milliliters of plasma every minute. It can directly expose the kidney to inflammatory mediators, which leads to the damage of renal tubular epithelial cells [7]. Histologically, renal tubular epithelial cells are vacuolated without the obvious apoptosis and necrosis [8]. Hypoxia in the hypoperfusion zone can further promote the inflammatory response of renal tubular cells. Then, the blood flow in this zone is also further slowed, which results in a long transport time of inflammatory mediators in the blood vessels, so the exposure of capillary endothelial cells and renal tubular epithelial cells to inflammatory mediators is further prolonged. Ultimately, the inflammatory response is amplified, thus triggering a stress response [9]. Hence, it is necessary to examine and diagnose renal function in AKI patients.

The article "Renal Doppler Ultrasound in the Evaluation of Renal Function in Patients with Sepsis" was retracted in 2023. Reasons: signs of a paper mill; compromised peer review; unreliable results or conclusions.

The renal Doppler ultrasound is a relatively mature technology, which is simple, economical, and non-invasive [10]. It can well determine the optimal mean artery pressure (MAP) for each patient [11]. Moreover, the renal Doppler ultrasound can not only detect renal morphological abnormalities but also provide qualitative or quantitative hemodynamic information of intrarenal or extrarenal vasculature. The renal resistance index (RRI) measured by Doppler ultrasound can accurately predict the occurrence of AKI [12]. RRI can be used as an independent predictor of acute and chronic kidney disease and renal failure [13]. The sensitivity of RRI during the progression of AKI is higher than the changes in serum creatinine (Cr) values in the recovering and developing regions [14]. To sum up, the renal Doppler ultrasound shows superior performance characteristics in distinguishing the transient AKI from persistent AKI, with a high value in evaluating renal function [15].

Patients with sepsis enrolled in the experiment were explored. Patients were classified into the AKI group and non-AKI group based on whether they had AKI. Renal Doppler ultrasound was performed on all patients to determine RRI and power Doppler ultrasound (PDU) scores. The differences of each index between the two groups were compared to provide a reference and basis for the diagnosis and treatment of related diseases in clinical practice.

## 2. Materials and Methods

### 2.1. Study Subjects

A total of 50 patients with sepsis or septic shock admitted to the hospital from February 2019 to March 2020 were selected. There were 28 male patients and 22 female patients, with a mean age of 55.3 ± 13.6 years. The patients were divided into AKI group (25 patients) and non-AKI group (25 patients) according to whether they had AKI. The experimental process had been approved by the ethics committee of hospital, and all subjects included in the study had signed the informed consent forms. Inclusion criteria: patients over 18 years old; patients who meet the diagnostic criteria of Sepsis 3.0 proposed by the European Society of Intensive Care Medicine (ESICM). Exclusion criteria: patients during pregnancy; patients with chronic renal insufficiency; patients with renal vascular disease; patients with obstructive renal failure; patients with arrhythmia; patients with hepatorenal syndrome.

The article "Renal Doppler Ultrasound in the Evaluation of Renal Function in Patients with Sepsis" was retracted in 2023. Reasons: signs of a paper mill; compromised peer review; unreliable results or conclusions.

### 2.2. Routine Processing

All patients underwent continuous monitoring of heart rate, finger oxygen saturation, blood pressure, and pulse pressure using multifunctional monitor, and hourly urine output was recorded. Patients' vasoactive and nephrotoxic drug use were recorded at the time of ultrasound. In addition, the injury severity score (ISS), acute physiology and chronic health evaluation II (APACHE II) 24 hours after admission to ICU, Glasgow coma scale (GCS), ICU length of stay (LOS), and duration of mechanical ventilation were recorded.

### 2.3. Methods of Renal Doppler Ultrasound

Renal Doppler ultrasound was performed 24 hours after admission to ICU under stable hemodynamic conditions. Color Doppler ultrasound diagnostic instrument was adopted, with a probe frequency of 4.0 MHz-5.5 MHz. Ultrasound needed to be performed daily for 7 days until the patient left the ICU. The ultrasound examination was performed by a physician trained in ultrasound in acute and critical illness who wasn't involved in the diagnosis and treatment of the patient and also wasn't aware of the patient's condition. Then, the filterable ultrasound was adopted to explore the kidney to check whether there was hematoma and contusion. Besides, the damage to the renal arteries was checked. Finally, the interlobular artery resistance index was measured. The right kidney was preferred. If the right kidney could not be measured, the left one was selected.  Figure 1 showed the measurement process.

Patients in the two groups received the PDU examination, and the images were stored. The PDU scoring was performed by another physician who specialized in critical illness.  Figure 2 showed the specific ultrasound images corresponding to each rating level, where the red spot represented the blood flow signal of the orientation probe, and the green box represented the blood flow signal area. The scoring method of PDU was as follows. 0 point meant that no renal vessels were detected, 1 point meant that there were few vessels at the hilum, 2 points meant that interlobar vessels were detected in most renal parenchyma, and 3 points meant that there was renal angiography at the arcuate artery level detected throughout the kidney.

The article "Renal Doppler Ultrasound in the Evaluation of Renal Function in Patients with Sepsis" was retracted in 2023. Reasons: signs of a paper mill; compromised peer review; unreliable results or conclusions.

### 2.4. Observation Indexes

Venous blood samples were collected, and creatinine (Cr), blood urea nitrogen (BUN), and C-reactive protein (CRP) were measured. Besides, a routine urine examination was performed. Arterial blood gas analysis was performed, and the serum creatine kinase (CK), serum cystatin C (Cys C), serum *β*2 microglobulin (*β*2-MG), and procalcitonin (PCT) were determined at 1, 3, 5, and 7 days. The partial pressure of oxygen (PaO_2_) and that of carbon dioxide (PaCO_2_) were measured and recorded at the most recent time when the patient began to receive the ultrasound. The Cr concentration was calculated by the end-point colorimetry, and its absorbance was measured at 510-520 nm. Centrifugation was performed at 3,500 r/min for 10 min. The upper serum was taken, and the serum BUN level was determined by the automatic biochemical analyzer. The CRP test was performed by an automatic specific protein instrument (Siemens BNII).

### 2.5. Diagnostic Criteria for AKI

The diagnosis was made according to the diagnostic criteria for AKI established by the 2012 Kidney Disease: Improving Global Outcomes (KDIGO), and AKI could be diagnosed if one of the following conditions was met: (1) renal function decreased dramatically within 48 hours, mainly manifested as an increase in serum creatinine (Scr) ≥26.5 *μ*mol/L. (2) Renal impairment within 7 days; Scr increased to ≥1.5 times the baseline value. (3) The urine volume was less than 0.5 mL/(kg·h) for more than 6 hours.

### 2.6. Data Analysis

SPSS 11.0 was employed for data statistics and analysis. The receiver operating characteristic (ROC) curves of RRI at different times were drawn to evaluate the diagnostic value of AKI. Measurement data were expressed as mean ± standard deviation ($\overset{¯}{\text{x}}$±s), and the *t*-test was used to test the significance of patient data before and after surgery. Enumeration data were expressed as actual number and percentage (%), *χ*^2^ test was adopted to test the significance, and *P <0.05* was considered statistically significant.

## 3. Results

### 3.1. Basic Data of Patients

Table 1 showed the basic data of patients. The ratio of males to females in the AKI group was 16 : 9, and the mean age was 50.1 ± 11.2 years old. The ratio of males to females in the non-AKI group was 14 : 11, and the mean age was 52.3 ± 13.6 years old. The difference between the two groups wasn't considerable (*P* >0.05), with comparability.

### 3.2. Comparison of RRI between the AKI Group and the Non- AKI Group

Figure 3 showed the changes in RRI in the AKI group and the non-AKI group. The RRI of 7 days in the AKI group was 0.71, 0.73, 0.72, 0.76, 0.76, 0.77, and 0.75. The RRI of 7 days in the non-AKI group was 0.63, 0.6, 0.62, 0.67, 0.7, 0.72, and 0.71. RRI in both groups showed a slight upward trend over time. From day 1 to day 7, the RRI of the AKI group was observably higher than that of the non-AKI group, with a considerable difference (*P* <0.05).

The article "Renal Doppler Ultrasound in the Evaluation of Renal Function in Patients with Sepsis" was retracted in 2023. Reasons: signs of a paper mill; compromised peer review; unreliable results or conclusions.

### 3.3. ROC Curve Analysis of RRI at Different Times for the Diagnosis of AKI

The results of ROC curve analysis of RRI at different times for the diagnosis of AKI were shown in Table 2. The areas under ROC curve of AKI group 7 days after admitted to ICU were 0.745, 0.683, 0.729, 0.856, 0.793, 0.819, and 0.836, respectively, and the difference had statistical meaning (*P <0.05*). The area under the ROC curve of RRI in the diagnosis of AKI at 1 to 7 days was compared pairwise using the Z test, and the comparison results are given in Figure 4. There was no significant difference in the area under ROC curve between the two groups at each time (*P >0.05*).

### 3.4. Comparison of PDU Scores between the AKI Group and the Non-AKI Group

Figure 5 showed the PDU scores of the two groups. In the two groups, the most people scored 2 points. With PDU score as the dependent variable, the grouping of AKI and the time as the fixed effect, and individual patients as the random effect, the linear model statistical analysis showed that there was no statistical difference between the two groups (*P* >0.05). There was a statistically insignificant difference in the RRI measured at different times within 7 days after admission to ICU between the two groups (*P* >0.05).

## 4. Discussion

The kidney is one of the most vulnerable organs in critically ill patients. Studies suggested that the probability of AKI in patients undergoing common surgery is only 1%, but the proportion in critically ill patients rises to 35%. AKI can slowly develop into chronic renal failure and eventually become an independent risk factor of death. Through cytokines, leukocyte vascular exudation, oxidative stress, sodium, and water channel regulation dysfunction, AKI can eventually lead to organ dysfunction. Although the renal function has been restored, the interaction of organ functions during AKI can lead to long-term complications in distant organs. Although organ support and rescue resuscitation techniques have been greatly improved, the incidence and mortality of AKI are still high. AKI can slowly develop into chronic renal failure and eventually become an independent risk factor for death. There are many factors that can trigger AKI such as hypovolemia, shock, major surgery, trauma, and heart failure [16], of which the most common factor is sepsis. According to some research, the mortality rate of patients with septic AKI is much higher than that of patients with AKI of other causes [17]. Moreover, the 90-day mortality rate of AKI in sepsis is as high as 50%-90% [18, 19]. AKI is one of the most universal organ dysfunction in sepsis that can increase the risk of adverse outcomes [20, 21]. RRT is the main treatment for sepsis-associated AKI [22, 23]. After the effects of early and delayed strategies on outcomes in ICU patients with sepsis-associated AKI were compared, Wu et al. (2020) found that early initiation of continuous renal replacement therapy (CRRT) in patients with sepsis-associated AKI could shorten the duration of CRRT [24]. Therefore, the early prediction and diagnosis of AKI had a positive value.

The article "Renal Doppler Ultrasound in the Evaluation of Renal Function in Patients with Sepsis" was retracted in 2023. Reasons: signs of a paper mill; compromised peer review; unreliable results or conclusions.

Most of the diagnostic grading criteria are based on Scr and urine volume. Cr and urine volume, as representative indexes, have a role in reflecting renal function [25]. Renal ultrasound is widely applied in the diagnosis of renal diseases because of its simplicity, rapidity, non-invasiveness, and economy [26]. The color Doppler ultrasound can achieve ideal diagnostic results through the changes of renal size, renal cortical thickness, and ultrasonic parameters [27]. The advantage of Doppler ultrasound lies not only in the examination of renal morphological abnormalities but also in the monitoring of renal function [28]. By detecting changes in intrarenal blood flow, the color Doppler, energy Doppler, and spectral analysis can provide qualitative or quantitative hemodynamic information about the intrarenal and extrarenal vasculature. Most of the renal parenchymal changes are related to the hemodynamics of the intrarenal artery. Renal Doppler ultrasound can well monitor the blood flow grading of patients [29]. RRI, renal pulse index, systolic peak flow velocity, acceleration time, and acceleration index are the commonly used quantitative parameters in renal flow Doppler waveform, especially RRI. This index can monitor renal perfusion in patients in real time, with good diagnosis and prediction effects on acute tubular necrosis, obstructive nephropathy, hepatorenal syndrome, and renal cell carcinoma [30]. For patients with sepsis or severe infection, the RRI of patients with AKI is markedly higher than that of patients without AKI [31]. Qin et al. (2019) analyzed the early prediction effect of Doppler RRI and semi-quantitative color (SQC) on postoperative AKI in patients with aortic dissection, and they found that both postoperative RRI and SQC Doppler grading were independent predictors of postoperative AKI in patients with aortic dissection [32]. Doppler ultrasound can quickly obtain the postoperative RRI and SQC Doppler grading, which is a good tool for early prediction of postoperative AKI.

The article "Renal Doppler Ultrasound in the Evaluation of Renal Function in Patients with Sepsis" was retracted in 2023. Reasons: signs of a paper mill; compromised peer review; unreliable results or conclusions.

Renal function was monitored in all patients by using the renal Doppler ultrasound in this experiment. The RRI and PDU scores were compared between patients with AKI and those without. The results showed that the RRI in both groups showed a slight upward trend with the time delay. The RRI of the AKI group was manifestly higher compared with the non-AKI group from day 1 to day 7, with a considerable difference (*P* <0.05). The differences in the area under the ROC curve of RRI at different times between the two groups were not statistically considerable (*P* >0.05). Besides, the number of people with 2 points in PDU score was the largest in the two groups. With PDU score as the dependent variable, the grouping of AKI and the time as the fixed effect, and individual patients as the random effect, the linear model statistical analysis showed there was no statistical difference between the two groups (*P* >0.05). Furthermore, there was no statistically considerable difference in the RRI measured at different times within 7 days after admission to ICU between the two groups (*P* >0.05), which was possibly related to the individual differences and disease differences among subjects.

## 5. Conclusion

The RRI and PDU scores were compared between AKI patients and non-AKI patients in this experiment. The results reflected that the RRI of patients in the AKI group was higher than that in the non-AKI group, and the difference in PDU scores wasn't considerable between the two groups (*P* >0.05). Consequently, the RRI had a high diagnostic value for AKI, while the PDU score had little. This work provided a new idea and reference for the clinical diagnosis and treatment of septic AKI. Nevertheless, there are some deficiencies. For instance, the observation time is only one week, and the related indexes of renal Doppler ultrasound before and after AKI and during recovery aren't investigated. In the future, these problems will be improved to verify the results.

## Figures and Tables

**Figure 1:** Flow chart of RRI measurement.

**Figure 2:** Ultrasound images corresponding to each grade of scoring. (a): 0 point; (b): 1 point; (c): 3 points; (d): 4 points.

**Figure 3:** Changes of RRI between the AKI group and the non-AKI group. ∗ meant that the differences between the groups were statistically considerable, *P <0.05*.

**Figure 4:** Area comparison under the ROC curve of RRI for AKI diagnosis at different times in ICU.

**Figure 5:** PDU scores of the AKI group and the non-AKI group. (A: AKI group; B: non-AKI group).

The article "Renal Doppler Ultrasound in the Evaluation of Renal Function in Patients with Sepsis" was retracted in 2023. Reasons: signs of a paper mill; compromised peer review; unreliable results or conclusions.

**Table 1:** Basic data of patients in the two groups.

Item	Non-AKI group (n =25)	AKI group (n =25)	Statistic (*χ*^2^ or *t*)	*P*
Gender [male: Female]	14 : 11	16 : 9	0.213	0.768
Age (years)	52.3 ± 13.6	50.1 ± 11.2	1.835	0.113
BMI	23.4 ± 3.3	21.5 ± 2.5	0.721	0.584
ISS	29.8 ± 7.7	30.6 ± 2.9	0.590	0.487
APECHE II	14.2 ± 9.1	16.3 ± 7.6	4.186	0.022
Glasgow coma index	16 (8 ~ 18)	14 (13~17)	0.108	0.533
Mechanical ventilation time (d)	7.8 ± 8.6	8.5 ± 11	0.715	0.632
ICU LOS (d)	11.3 ± 9.9	12.02 ± 8.6	0.789	0.523
Mortality (cases)	8	12	11.328	≤0.001

**Table 2:** Area under the ROC curve analysis of RRI for the diagnosis of AKI at different times of ICU admission.

Time	Area under the ROC curve	95% CI	*P*
Day 1	0.745	0.624 (0.513~0901)	0.038
Day 2	0.683	0.548 (0.437~0.916)	0.019
Day 3	0.729	0.611 (0.547~0.869)	0.007
Day 4	0.856	0.538 (0.469~0.937)	0.037
Day 5	0.793	0.637 (0.469~0.873)	0.021
Day 6	0.819	0.463 (0.411~0.943)	0.016
Day 7	0.836	0.672 (0.501~1.000)	0.036

## Data Availability

The data used to support the findings of this study are available from the corresponding author upon request.
